The article "Uncertainty Estimation Using Variational Mixture of Gaussians Capsule Network for Health Image Classification" was published in 2022. Journal: Comput Intell Neurosci.

# Uncertainty Estimation Using Variational Mixture of Gaussians Capsule Network for Health Image Classification

**DOI:** 10.1155/2022/4984490

**Published:** 2022-09-30

**Authors:** Patrick Kwabena Mensah, Mighty Abra Ayidzoe, Alex Akwasi Opoku, Kwabena Adu, Benjamin Asubam Weyori, Isaac Kofi Nti, Peter Nimbe

**Affiliations:** ^1^Department of Computer Science and Informatics, University of Energy and Natural Resources, P. O. Box 214, Sunyani, Ghana; ^2^Department of Mathematics and Statistics, University of Energy and Natural Resources, P. O. Box 214, Sunyani, Ghana; ^3^School of Information Technology, University of Cincinnati, OH, USA

## Abstract

Capsule Networks have shown great promise in image recognition due to their ability to recognize the pose, texture, and deformation of objects and object parts. However, the majority of the existing capsule networks are deterministic with limited ability to express uncertainty. Many of them tend to be overconfident on out-of-distribution data, making them less trustworthy and hence reducing their suitability for practical adoption in safety-critical areas such as health and self-driving cars. In this work, we propose a capsule network based on a variational mixture of Gaussians to train distributions of network weights as opposed to a single set of weights and enable the model to express its predictive uncertainty on out-of-distribution data. Training distributions of weights have the added advantage of avoiding overfitting on smaller datasets which are common in health and other fields. Although Bayesian neural networks are known to exhibit slow training and convergence, experimental results show that the proposed model can retrieve only relevant features, converge faster, is less computationally complex, can effectively express its predictive uncertainties, and achieve performance values that are comparable to the state-of-the-art models. This is an indication that CapsNets can exhibit the transparency, credibility, reliability, and interpretability required for practical adoption.

## 1. Introduction

Recently, there has been an upsurge in the adoption of Deep Learning (DL) to perform complex tasks such as Visual Question Answering [1], and plant disease detection [2], among others, due to their excellent performance in terms of speed and accuracy compared to humans. Capsule Networks [3, 4], for example, have demonstrated the ability to recognize the pose, texture, and deformation of an object and its parts. They have thus been proposed for use in sensitive areas such as health [5, 6] and agriculture [7, 8], among others. Irrespective of the sensitivity of the application area, capsule networks (just like many other deep learning models) do not incorporate uncertainties in their predictions. The inability to model uncertainties leads to model over/under confidence [9]. We propose a Bayesian Capsule Network (BCN) motivated by [10, 11] and on the background that the Bayesian framework provides the capability for modeling uncertainties in neural network predictions [12]. Bayesian Neural Networks (BNNs) estimate uncertainties by defining a distribution over the network weight parameters whose posterior weight distribution *p*(.*|x*) permits the BNN to capture the prediction uncertainties.

BNNs are known to have a longer convergence time during training [11] since training occurs on larger distribution parameters compared to single points in deterministic models. However, the choice of appropriate normalization and weight initialization schemes can allow the network to converge faster. Since Bayesian models replace the fixed weights with probability distributions, they are capable of training on smaller datasets without overfitting.

This work, therefore, proposes a Variational Mixture of Gaussian-based capsule network (CapsNet) that will contribute to solving problems such as those caused by the lack of huge datasets in critical areas (e.g., in health). Additionally, we aim at reducing model complexity, reducing convergence time, and improving accuracy on difficult datasets that are small and imbalanced. These are difficult targets for a Bayesian model known for its complexity, and inability to converge faster to achieve. We also aim to leverage the ability of the BNN to model uncertainties and introduce some form of reliability in the predictions of the model on input images. The motive is to enable such models to gain the confidence of the practitioner for practical adoption in safety-critical areas such as autonomous cars and medicine. The lack of sufficient training data is a major limiting factor to the adoption of deep learning in areas such as health due to concerns related to overfitting. This work, therefore, uses Bayesian NNs to elegantly avoid this problem by acting on the distributions weights as opposed to deterministic models which train on a single set of weights. For instance, the parameter *θ* of a distribution on the weights *p*(*w|θ*) is learned by Variational Inference leading to the minimization of Kullback–Leibler (KL) divergence. This method provides a principled framework for the usage of model components leading to better monitoring of model complexity and avoiding its associated problems such as overfitting. In addition, regularization is natural to BNNs such that the regularization parameters get consistent treatment in the Bayesian setting thus eliminating the need for techniques such as cross-validation [13]. Perhaps, one of the main benefits of our method to the health and other critical sectors is the model's ability to avoid overconfident predictions in regions of sparse data.

Experimental results show that our proposed Variational Mixture of Gaussians Routing (VMGs-Routing) achieves a significant reduction in model complexity while achieving competitive results compared to the state-of-the-art models. Our routing algorithm improves upon similar existing routing algorithms by training and learning faster to achieve convergence within a few epochs (approximately 100 epochs). This method further reduces the infinite likelihood and zero variance problem inherent in Maximum Likelihood solutions caused by Gaussian clusters that try to take sole possession of data points (also known as polarization in Capsules).

The contributions of this paper can be summarized as follows:

1. We propose a routing method from a variational mixture of Gaussians that clearly relies on the maximization of the evidence lower bound (ELBO) to activate a capsule.
2. We provide empirical results that are comparative to state-of-the-art previous works on Bayesian and deterministic capsules to demonstrate that our approach does not result in the loss of any of the inherent strengths of capsules such as viewpoint-invariance, robustness.
3. We show that our proposed Bayesian CapsNet is not overconfident and is reliable from the high uncertainty it expresses on out-of-distribution data.
4. The proposed model is less computationally complex and performs comparatively well with deep Bayesian CapsNet models from the literature in terms of accuracy, uncertainty estimation, and prediction. Comparatively, our model achieves better speedup during training and testing without performance degradation.
5. We provide extensive visualizations of layer activation maps, and predictive uncertainty plots, among others in an attempt to increase the interpretability of our model which is presumed (as a Bayesian model) to be a complex probabilistic ‘black box' model.

The rest of the paper is organized in the following way: Section 2 presents the related works in the literature followed by Section 3 which discusses the Bayesian methods adopted for this work.  Section 4 presents the experiments and experimental results after which the paper is concluded in Section 5.

## 2. Related Work

Some works in the literature have relied on variational inference to propose capsules to solve varied problems. Smith et al. [14] proposed a probabilistic capsule (CapsNet) to encode the capsule assumptions and separate the generative and inference parts from each other. They showed that their model can generalize well on out-of-distribution data, but did not express the uncertainty of their model. Ribeiro et al. [11] proposed a Bayesian CapsNet routing algorithm based on a mixture of transforming Gaussians to address the variance collapse problem and to model the uncertainty of the pose parameters. However, experimental results of the uncertainty of the pose parameters were not provided. In this implementation, a parent capsule *j* is activated if there is an agreement between the votes of adjacent capsules. The agreement is measured by the entropy of the multivariate Gaussian distribution. A conditional variational CapsNet [15] was proposed to detect classes that are not known during training as a contribution to the open set recognition problem. To this end, they adopted the variational autoencoder approach enabling similar features to assume the shape of a Gaussian, such that each unique feature assumed a different Gaussian. A flow-based model with a long flow structure is capable of finding the approximate posterior probability compared to utilizing a simple family of distributions to approximate the intractable posterior. However, as the data increase in dimensionality, this solution gives rise to huge computational complexity and variance. To address this shortcoming, Hua et al. [16] utilized a dynamic routing flow with variational inference to achieve a shorter flow structure and a significant improvement in precision and accuracy. To introduce routing uncertainties in CapsNet, Ribeiro et al. [17] proposed a global view of the local iterative routing between capsules of adjacent layers, enabling them to capture the uncertainty in the assignment of parts to objects. Compared to the two previous works mentioned earlier, this partial Bayesian CapsNet produced results on out-of-distribution predictive entropies that were consistent with uncertainties of model predictions. To avoid the singularity problem caused by maximum likelihood estimation (MLE), a variational routing CapsNet [18] has been proposed to utilize the variational distribution and integrate the prior distribution for automatic determination of the class of data and avoid overfitting. A Bayesian capsule encoder [19] was proposed to regulate the standard deviation and mean in latent space. The authors argue that it is a better approach for the retrieval of relevant features and image reconstruction from latent space. To demonstrate that deep variational CapsNets can achieve better performance on image synthesis and analysis, Huang et al. [20] proposed a variational model in which the divergence between a capsule and a given prior distribution defines the presence of different entities in an object.

Traditionally, uncertainty is modeled with probability theory and is increasingly becoming more relevant due to the adoption of deep learning (DL) models in practical and safety-critical applications such as medicine and self-driving cars. This type of modeling uses a single probability distribution to capture the required knowledge and struggles to express the two types of uncertainties in a DL model [21]. Aleatoric uncertainty arises from the element of randomness due to the variability of the outcome of events, while epistemic uncertainty measures the modeler(s) inability to design the best model for the task at hand. In the literature, Bayesian networks with latent variables have been proposed [22] to measure both the predictive aleatoric and epistemic uncertainties. This approach played a significant role in the interpretability of the model, which, like other neural network models is perceived to be a “black box.” With the inherent advantages of CapsNets over other neural networks, our work proposes a variational mixture of Gaussians routing-based capsules to effectively capture the predictive uncertainty on the in and out-of-distribution data to improve reliability, interpretability, and model confidence for safety-critical applications.

## 3. Proposed Methods

In this section, we outline a brief introduction to the concepts of Variational Inference and Gaussian mixture models on which our routing algorithm is based.

### 3.1. Bayesian Mixture of Gaussians

Suppose *X* assumes a Gaussian distribution; a linear combination of these Gaussians forms the basis for the formulation of a mixture of probabilistic (Gaussian) models known as a mixture of Gaussians [10]. This convex combination creates the opportunity to adjust the means, covariances, and coefficients as a basis for approximating any continuous density function to arbitrary accuracy. Considering a superposition of K-Gaussian densities taking the form of the joint probability *p*(*x*, *z*) = *p*(*x|z*)*p*(*z*), *z* can be marginalized out to give *p*(*x*) = ∑_*z*=1_^*K*^*p*(*x*, *z*) = ∑_*z*=1_^*K*^*p*(*z*)*p*(*x|z*). Realizing that the mixing coefficient *π*_*z*_ = *p*(*z*) = 1/*K* (*K* is a one-hot-vector) is the probability of choosing one cluster out of *K* clusters, the marginal probability can be rewritten in the form of a Gaussian Mixture Model (GMM), shown in equation (1):

(1) $$\begin{array}{c} p\left(x\right)=\sum_{k=1}^{K}\pi_{z}N\left(x_{i}|\mu_{k},\Sigma_{k}\right). \end{array}$$

The Gaussian density (also called component) in the above expression has its own mean *μ*_*k*_ and covariance Σ_*k*_.

Since routing in capsules operates on the concept of clustering, they can naturally be modeled via a mixture of transforming Gaussians [11].

### 3.2. Variational Bayes

Bayesian algorithms perform inference on unknown random variables by finding a posterior probability density [23] in situations where the posterior is intractable to compute. Approximate inference (using Variational Inference (VI)) provides a reasonable approximation to the problem compared to Markov Chain Monte Carlo (MCMC) methods that provide an exact solution but with slow convergence time.

Using the Bayes theorem, the posterior probability density can be computed as follows:

(2) $$\begin{array}{c} p\left(\vartheta |x\right)=\frac{p\left(\vartheta ,x\right)}{p\left(x\right)}\\ =\frac{p\left(x|\vartheta \right)p\left(\vartheta \right)}{p\left(x\right)}\\ =\frac{p\left(x|\vartheta \right)p\left(\vartheta \right)}{\int_{\vartheta }p\left(x,\vartheta \right)d\vartheta }, \end{array}$$

where ∫_*θ*_*p*(*x*, *ϑ*)d*ϑ* is the marginal probability (also called the evidence). This term is intractable, requiring the use of approximate solutions such as VI. VI does this by searching a family of distributions *Q* for the distribution *q* that is closest to the posterior *p*(.*|x*). The distance between the variational (“*nice*”) distribution *q* and the true posterior *p*(.*|x*); is measured by the Kullback–Leibler (KL) divergence.

(3) $$\begin{array}{c} KL\left[q\|p\left(.|x\right)\right]=\int q\left(\vartheta \right)\log\frac{q\left(\vartheta \right)}{p\left(\vartheta |x\right)}d\vartheta \\ =E_{q}\log\frac{q\left(\vartheta \right)}{p\left(\vartheta |x\right)}\\ =\log p\left(x\right)-\int q\left(\vartheta \right)\log\frac{p\left(x,\vartheta \right)}{\;q\left(\vartheta \right)}\text{d}\vartheta . \end{array}$$

Therefore, minimization of the KL over *q* now becomes maximization of the Evidence Lower Bound (ELBO)

(4) $$\begin{array}{c} \text{ELBO}=ℒ\left[q\right]\left(x\right)\\ =\int q\left(\vartheta \right)\text{log}\frac{p\left(x,\vartheta \right)}{q\left(\vartheta \right)}\text{d}\vartheta , \end{array}$$

to avoid the intractability issues of the true posterior *p*(*ϑ|x*). To maximize the ELBO, the vector of hidden random variables *θ*=(*θ*_1_, *θ*_2_,…, *θ*_*n*_) (distributed according to the variational distribution  *q*) are assumed to be made up of independent random variables allowing their joint distribution to be obtained from the product of their marginal distributions.

(5) $$\begin{array}{c} q\left(\theta \right)=q\left(\theta_{1},\theta_{2\;},\ldots \theta_{n}\right)\\ =\prod_{i=1}^{n}q_{i}\left(\theta_{i}\right). \end{array}$$

This mean-field (MF) approximation makes it possible to obtain a free-form optimization of the ELBO ℒ[*q*] with respect to all the distributions *q*_*i*_(*θ*_**i**_) by optimizing each of the factors in turn. When the ℒ[*q*] is fully described by the MF distribution, every data point described by a variational distribution will have its own free parameters. The task is to then find the free parameters that will maximize ℒ[*q*].

In this study, it is assumed that data points, which are the realization of the random variables *X*_*1*_ ,…, *X*_*N*_, are taken from the *m*-dimensional Euclidean space *R*^*D*^. Thus, the dataset *X* = (*X*_1_,…, *X*_*N*_) is a vector with *R*^*D*^-valued random coordinates that are to be classified into *K* clusters with random centroids *H*_*1*_*,…, H*_*K*_ that are multinormally distributed, i.e., *H*_*k*_*∼N*(*μ*_*k*_, Δ_*k*_^−1^), where *k* = 1,.., *K,μ*_**k**_ is the 1 × D mean-vector and Δ_**k**_^−1^ the *D* × *D* covariance matrix. In what follows, *f*_*k*_ will be written for the density of *N*(*μ*_*k*_, Δ_*k*_^−1^). Whenever the random variable *X*_*n*_ is in the *k*^*th*^ cluster, it then assumes the distribution of the centroid of that cluster. Thus, each data point *X*_*n*_ is distributed according to *N*(*μ*_*k*_, Δ_*k*_^−1^), for some = 1,.., *K.* In the sequel we denote by *C*_*n*_, the cluster label of the random variable *X*_*n*_, for *n* = 1,*…, N.* To each data point *X*_*n*_, corresponds a latent variable *Z*_*n*_, that is a 1-of-*K* binary vector with π_*k*_ being the probability *Z*_*nk*_ = 1, for some *k* = 1,.., *K.* Therefore, π =  (π_1_,…, π_*K*_), called the vector of mixing coefficients, is a probability vector and *N* *=* (*N*_1_,…, *Y*_*K*_) = *Z*_*1*_ *+* *Z*_*2*_*+ … + Z*_*N*_ is a random vector with *K* non-negative coordinates that sum up to *N.* In fact, *Y* is multinomially distributed with parameters N and π. Observe that for any *n* = 1,…, N, the probability that *Z_n_* = *z_n_* is given by the following equation:

(6) $$\begin{array}{c} p\left(z_{n}\right)=\prod_{k=1}^{K}\pi_{k}^{z_{nk}}. \end{array}$$

Putting *θ* = (*Z*, π, *μ*,Λ), with *Z* = (Z_1_,…, Z_N_), *μ* = (*μ*_1_, *μ*_2_,…, *μ*_K_) and Λ = (Λ _1_, Λ _2_,…, Λ _K_), the joint distribution of *X* and *θ* can be written as follows:

(7) $$\begin{array}{c} p\left(X,\theta \right)=p\left(X|Z,\mu ,\Lambda \right)p\left(Z|\pi ,\mu ,\Lambda \right)p\left(\pi |\mu ,\Lambda \right)p\left(\mu |\Lambda \right)p\left(\Lambda \right)\\ =p\left(X|Z,\mu ,\Lambda \right)p\left(Z|\pi \right)p\left(\pi \right)p\left(\mu |\Lambda \right)p\left(\Lambda \right). \end{array}$$

The second equality of equation (7) uses that *p*(*Z|π*, *μ*, Λ) = *p*(*Z|π*) and *p*(*π|μ*, *π*) = *p*(*π*). We assume further that conditioning on *θ*, the components of *X* are independent. Similarly, given *π* and Λ, the components of *Z* and *μ* are respectively independent. Furthermore, the components of Λ are also independent. In addition to the above prescription, we use the plate notation (directed graph) [10, 24] to derive our priors and put the problem in a Bayesian setting. Thus, using the conjugate priors of , *Λ* and *π*, and the above-given result in

(8) $$\begin{array}{c} \pi ∼\text{SymDir}\left(K,\propto_{0}\right),\\ \Lambda_{k=1,\ldots ,K}∼Wi\left(W_{0},v_{0}\right),\\ \mu_{k=1,\ldots ,K}∼N\left(\left(\mu_{0}\right),{\left(\beta_{0}\Lambda_{k}\right)}^{-1}\right),\\ Y=\left(Y_{1},\ldots ,Y_{K}\right)∼\text{Mult}\left(N,\pi \right),\\ X_{i=1,\ldots ,N}∼N\left(\mu_{C_{i}},\Lambda_{C_{i}}^{-1}\right), \end{array}$$

Therefore,

(9) $$\begin{array}{c} p\left(x|z,\mu ,\Lambda \right)=\prod_{n=1}^{N}\prod_{k=1}^{K}f_{k}{\left(x_{n}\right)}^{z_{nk}}, \end{array}$$

(10) $$\begin{array}{c} p\left(z|\pi \right)=\prod_{n=1}^{N}\left(\prod_{k=1}^{K}{\left(\pi_{k}\right)}^{z_{nk}}\right), \end{array}$$

(11) $$\begin{array}{c} p\left(\pi \right)=\frac{\Gamma \left(K\propto_{0}\right)}{\Gamma {\left(\propto_{0}\right)}^{K}}\prod_{k=1}^{K}\pi_{k}^{\alpha_{0}-1}, \end{array}$$

(12) $$\begin{array}{c} p\left(\mu |\Lambda \right)=\prod_{k=1}^{K}f_{k}^{0}\left({µ}_{k}\right), \end{array}$$

(13) $$\begin{array}{c} p\left(\Lambda \right)=\prod_{k=1}^{K}Wi\left(\Lambda_{k}\right), \end{array}$$

where

(14) $$\begin{array}{c} f_{k}\left(x_{n}\right)=\frac{1}{2\pi^{D/2}}\frac{1}{{\left|\Lambda_{k}^{-1}\right|}^{1/2}}\text{exp}\left\{-\frac{1}{2}{\left(x_{n}-\mu_{k}\right)}^{T}\Lambda_{k}\left(x_{n}-\mu_{k}\right)\right\},\\ f_{k}^{0}\left(\mu_{k}\right)=\frac{1}{2\pi^{D/2}}\frac{1}{{\left|{\left(\beta_{0}\Lambda_{k}\right)}^{-1}\right|}^{1/2}}\text{exp}\left\{-\frac{1}{2}{\left(\mu_{k}-\mu_{0}\right)}^{T}\beta_{0}\Lambda_{k}\left(\mu_{k}-\mu_{0}\right)\right\},\\ Wi\left(\Lambda_{k}\right)=B\left(W_{0},v_{0}\right){\left|\Lambda_{k}\right|}^{\left(v_{0}-D-1\right)/2}\text{exp}\left(-\frac{1}{2}Tr\left(W_{k}^{-1}\Lambda_{k}\right)\right),\\ B\left(W_{0},v_{0}\right)={\left|W_{0}\right|}^{-v_{0}/2}{\left\{2^{v_{0}D/2}\pi^{D\left(D-1\right)/4}\prod_{\text{i}=1}^{D}\Gamma \left(\frac{v_{0}+1-i}{2}\right)\right\}}^{-1}. \end{array}$$

From the joint distribution in (7), we identify the posterior and variational (‘*nice'*) distributions as *p* (*Z*, *μ*, *Λ*, *π|*X) and *q*(*Z*, *μ*, Λ, *π*) i.e., the *p*(*θ|X*) and *q*(*θ*) respectively, providing the ingredients for the computation of *KL*[*q*(*Z*, *μ*, Λ, *π*)*‖p*(*Z*,  *μ*, Λ, *π|X*)]. Accordingly, the variational distribution (VD) is factorized based on the MF approximation method to obtain *q*(Z, *μ*, *Λ*, *π*) = *q*(Z)*q*(*μ*, *Λ*, *π*). Meanwhile, from the MF approximation, it can be shown that the best distribution *q*_*j*_ for maximizing the ELBO is *q*_*j*_^*∗*^(.*|x*), satisfying ln*q*_*j*_^*∗*^(*z|x*) = ln*p*(*z*_*j*_, *x*) + constant. We consequently model the joint distribution in (7) according to the aforementioned best variational distribution. Initial calculations involve the determination of *q*^*∗*^(*z|x*) followed by *q*^*∗*^(*π*, *μ*, Λ). In other words,

(15) $$\begin{array}{c} log\;q^{*}\left(z|x\right)=E_{q\left(\pi ,\mu ,\Lambda \right)}\left[\log\left(p\left(x|z,\mu ,\Lambda \right)p\left(z|\pi \right)p\left(\pi \right)p\left(\mu ,\Lambda \right)\right)\right]+\text{const.} \end{array}$$

Pushing the variables not dependent on *z* (i.e. *p*(*π*)*p*(*μ*, Λ)) into the constant, we obtain the following equation:

(16) $$\begin{array}{c} log\;q^{*}\left(z|x\right)=E_{q\left(\pi ,\mu ,\Lambda \right)}\left[\log\left(p\left(x|z,\mu ,\Lambda \right)p\left(z|\pi \right)\right)\right]+\text{const} \end{array}$$

Substituting (9) and (10) into the expression for log *q*^*∗*^(*z|x*), produces

(17) $$\begin{array}{c} log\;q^{*}\left(z|x\right)=\sum_{n=1}^{N}\sum_{k=1}^{K}z_{nk}\text{log}\left(\rho_{nk}\left(x_{n}\right)\right)+\text{const}, \end{array}$$

where

(18) $$\begin{array}{c} log\rho_{nk}\left(x_{n}\right)=E_{q\left(\pi \right)}\left[\log\left(\pi_{k}\right)\right]-\frac{1}{2}E_{q\left(\pi \right)}\left[\log\left(\left|\Lambda_{k}^{-1}\right|\right)\right]\\ -\frac{D}{2}\log\left(2\pi \right)-\frac{1}{2}E_{q\left(\mu_{k},\Lambda_{k}\right)}\left[{\left(x_{n}-\mu_{k}\right)}^{T}\Lambda_{k}\left(x_{n}-\mu_{k}\right)\right]. \end{array}$$

Exponentiating log*q*^**∗**^(*z|x*) and normalizing it to let *ρ*_*nk*_ sum to 1 over all the values of *k* produces

(19) $$\begin{array}{c} q^{*}\left(z|x\right)=\prod_{n=1}^{N}\prod_{k=1}^{K}r_{nk}^{z_{nk}}\left(x_{n}\right), \end{array}$$

where

(20) $$\begin{array}{c} r_{nk}\left(x_{n}\right)=\frac{\rho_{nk}\left(x_{n}\right)}{\sum_{j=1}^{K}\rho_{nj}\left(x_{n}\right)}. \end{array}$$

The best *q*^*∗*^(*z|x*), therefore, is a product of categorical distributions for each latent variable having *r*_*nk*_ for *k*=1,2,…, *K* as parameters.

On the other hand, the best variational distribution *q*^*∗*^(*π*, *μ*, Λ) can be divided into two components *q*^*∗*^(*π*) and *q*^*∗*^(*μ*, *Λ*). It follows from the product rule, the deductions leading to equations (15), (9) and (10) that *q*^*∗*^(*π*) satisfies

(21) $$\begin{array}{c} \log q^{*}\left(\pi \right)=\log p\left(\pi \right)+E_{q\left(z\right)}\left[\log p\left(z|\pi \right)\right]+\text{const}\\ =\left(\alpha_{0}-1\right)\sum_{k=1}^{K}\ln\pi_{k}+\sum_{n=1}^{N}\sum_{k=1}^{K}z_{nk}\ln\pi_{k}+\text{const}\\ =\left(\alpha_{0}-1\right)\sum_{k=1}^{K}\ln\pi_{k}+\sum_{k=1}^{K}y_{k}\ln\pi_{k}+\text{const}. \end{array}$$

Taking exponentials of both sides of the above expression and taking care of the normalizing term result in

(22) $$\begin{array}{c} q^{*}\left(\pi \right)=\text{Dir}\left(K,\alpha_{1},\ldots ,\alpha_{K}\right)\\ =C\left(\alpha_{1},\ldots ,\alpha_{K}\right)\prod_{k=1}^{K}\pi_{k}^{\alpha_{k}-1}, \end{array}$$

where

(23) $$\begin{array}{c} \alpha_{k}=\alpha_{0}+y_{k}\text{ and}\\ y_{k}=\sum_{n=1}^{N}z_{nk}. \end{array}$$

Upon some computations, the variational distribution *q*^*∗*^(*μ*, *Λ*) for the joint distribution *q*(*μ*, *Λ*) takes the form

(24) $$\begin{array}{c} \log\left(q^{*}\left(\mu ,\Lambda \right)\right)=\log\left(p\left(\mu ,\Lambda \right)\right)+E_{q\left(z\right)}\left[\log\left(p\left(x|z,\mu ,\Lambda \right)\right)\right]+\text{const}\\ =\sum_{k=1}^{K}\left[\log\left(f_{k}^{0}\left(\mu_{k}\right)\right)+\log\left(Wi\left(\Lambda_{k}\right)\right)\right]+\text{const}, \end{array}$$

where *f*_*k*_^0^ and *Wi* are respectively the Gaussian and Wishart densities (see equations (12) and (13)) with parameters *m*_*k*_, *β*_*k*_, *W*_*k*_, and *v*_*k*_. These parameters are given as follows:

(25) $$\begin{array}{c} \beta_{k}=\beta_{0}+y_{k},\\ m_{k}=\frac{1}{\beta_{k}}\left(\beta_{0}\mu_{0}+y_{k}{\bar{x}}_{k}\right),\\ W_{k}^{-1}=W_{0}^{-1}+y_{k}S_{k}+\frac{\beta_{0}y_{k}}{\beta_{0}+y_{k}}\left({\bar{x}}_{k}-\mu_{0}\right){\left({\bar{x}}_{k}-\mu_{0}\right)}^{T},\\ v_{k}=v_{0}+y_{k},\\ y_{k}=\sum_{n=1}^{N}z_{nk},\\ {\bar{x}}_{k}=\frac{1}{y_{k}}\sum_{n=1}^{N}z_{nk}x_{n},\\ S_{k}=\frac{1}{y_{k}}\sum_{n=1}^{N}z_{nk}\left(x_{n}-{\bar{x}}_{k}\right){\left(x_{n}-{\bar{x}}_{k}\right)}^{T}. \end{array}$$

To evaluate *r*_*nk*_, the quantities in *ρ*_*nk*_ are expressed as follows:

(26) $$\begin{array}{c} E_{q^{*}\left(\mu_{k},\Lambda_{k}\right)}\left[{\left(x_{n}-\mu_{k}\right)}^{T}\Lambda_{k}\left(x_{n}-\mu_{k}\right)\right]=D\beta_{k}^{-1}+v_{k}{\left(x_{n}-m_{k}\right)}^{T}W_{k}\left(x_{n}-m_{k}\right),\\ \ln{\tilde{\Lambda }}_{k}\equiv E\left[\ln\left|{\tilde{\Lambda }}_{k}\right|\right]=\sum_{i=1}^{D}\psi \left(\frac{v_{k}+1-i}{2}\right)+D\ln2+\ln\left|W_{k}\right|,\\ \ln{\tilde{\pi }}_{k}\equiv E\left[\ln\left|\pi_{k}\right|\right]=\psi \left(\alpha_{k}\right)-\psi \left(\sum_{i=1}^{K}\alpha_{i}\right), \end{array}$$

where *ψ* is the log derivative of the multinomial gamma function.

After the substitutions, *ρ*_*nk*_ becomes,

(27) $$\begin{array}{c} ln\rho_{nk}=\left[\psi \left(\alpha_{k}\right)-\psi \left({\hat{\alpha }}_{k}\right)\right]+\frac{1}{2}\left[\sum_{i=1}^{D}\psi \left(\frac{\nu_{k}+1-i}{2}\right)+Dln2+ln\left|W_{k}\right|\right]\\ -\frac{D}{2}\ln\left(2\pi \right)-\frac{1}{2}\left[D\beta_{k}^{-1}+\nu_{k}{\left(x_{n}-m_{k}\right)}^{T}W_{k}\left(x_{n}-m_{k}\right)\right],\\ ln\rho_{nk}=\psi \left(\alpha_{k}\right)-\psi \left({\hat{\alpha }}_{k}\right)+\frac{1}{2}\sum_{1=1}^{D}\psi \left(\frac{\nu_{k}+1-i}{2}\right)+\frac{1}{2}Dln2\\ +\frac{1}{2}ln\left|W_{k}\right|-\frac{D}{2}\ln\left(2\pi \right)-\frac{1}{2}D\beta_{k}^{-1}-\frac{1}{2}\nu_{k}{\left(x_{n}-m_{k}\right)}^{T}W_{k}\left(x_{n}-m_{k}\right), \end{array}$$

where $\sum_{i=1}^{K}\alpha_{i}={\hat{\alpha }}_{i}$. There is a circular dependency between these variational parameters requiring *n* iterative updates that ensure the algorithm converges to an approximate posterior.

Using equation (7), the ELBO for a VGM model is obtained as follows:

(28) $$\begin{array}{c} ℒ=E\left[\text{In }p\left(X,Z,\pi ,\mu ,\Lambda \right)\right]-E\left[\text{In }q\left(Z,\pi ,\mu ,\Lambda \right)\right]. \end{array}$$

Applying the product rule, we obtain the following equation:

(29) $$\begin{array}{c} ℒ=\left\{E\left[\ln p\left(X|Z,\mu ,\Lambda \right)\right]+E\left[\ln p\left(Z|\pi \right)\right]+E\left[\ln p\left(\pi \right)\right]+E\left[\ln p\left(\mu ,\Lambda \right)\right]\right\}\\ -\left\{E\left[\ln q\left(Z\right)\right]-E\left[\ln q\left(\pi \right)\right]-E\left[\ln q\left(\mu ,\Lambda \right)\right]\right\}, \end{array}$$

and substituting the following expressions,

(30) $$\begin{array}{c} E\left[\ln p\left(X|Z,\mu ,\Lambda \right)\right]=\frac{1}{2}\overset{K}{\underset{k=1}{\sum }}Y_{k}\left\{\ln{\tilde{\Lambda }}_{k}-D\beta_{k}^{-1}-\nu_{k}Tr\left(S_{k}W_{k}\right)-\nu_{k}{\left(\bar{x_{k}}-m_{k}\right)}^{T}W_{k}\left(\bar{x_{k}}-m_{k}\right)-D\text{ln}\left(2\pi \right)\right\},\\ E\left[\ln p\left(Z|\pi \right)\right]=\overset{N}{\underset{n=1}{\sum }}\overset{K}{\underset{k=1}{\sum }}z_{nk}ln{\tilde{\pi }}_{k},\\ E\left[\ln p\left(\pi \right)\right]=\ln C\left(\alpha_{0}\right)+\left(\alpha_{0}-1\right)\sum_{k=1}^{K}\ln{\tilde{\pi }}_{k},\\ E\left[\ln p\left(\mu ,\Lambda \right)\right]=\frac{1}{2}\overset{K}{\underset{k=1}{\sum }}\left\{Dln\left(\frac{\beta_{0}}{2\pi }\right)+ln{\tilde{\Lambda }}_{k}-\frac{D\beta_{0}}{\beta_{k}}-\beta_{0}v_{k}{\left(m_{k}-m_{0}\right)}^{T}W_{k}\left(m_{k}-m_{0}\right)\right\}\\ +K\text{ln}B\left(W_{0},v_{0}\right)+\frac{\left(v_{0}-D-1\right)}{2}\overset{K}{\underset{k=1}{\sum }}ln{\tilde{\Lambda }}_{k}-\frac{1}{2}\overset{K}{\underset{k=1}{\sum }}v_{k}Tr\left(W_{0}^{-1}W_{k}\right),\\ E\left[\ln q\left(Z\right)\right]=\overset{N}{\underset{n=1}{\sum }}\overset{K}{\underset{k=1}{\sum }}z_{nk}\text{ln}r_{nk},\\ E\left[\ln q\left(\pi \right)\right]=\overset{K}{\underset{k=1}{\sum }}\left(\alpha_{k}-1\right)\ln{\tilde{\pi }}_{k}+\ln C\left(\alpha \right), \end{array}$$

and

(31) $$\begin{array}{c} E\left[\ln q\left(\mu ,\Lambda \right)\right]=\overset{K}{\underset{k=1}{\sum }}\left\{\frac{1}{2}\ln{\tilde{\Lambda }}_{k}+\frac{D}{2}\ln\left(\frac{\beta_{k}}{2\pi }\right)-\frac{D}{2}-ℋ\left[q\left(\Lambda_{k}\right)\right]\right\}, \end{array}$$

where ℋ[*q*(Λ_*k*_)] is the entropy of the Wishart distribution. **ℒ** then becomes the objective function to maximize and is given by the following equation:

(32) $$\begin{array}{c} ℒ=\left[\frac{1}{2}\sum_{k=1}^{K}Y_{k}\left\{ln{\tilde{\Lambda }}_{k}-D\beta_{k}^{-1}-\upsilon_{k}T_{r}\left(S_{k}W_{k}\right)-\upsilon_{k}{\left({\bar{x}}_{k}-m_{k}\right)}^{T}W_{k}\left({\bar{x}}_{k}-m_{k}\right)-Dln\left(2\pi \right)\right\}\right]\\ +\left[\sum_{n=1}^{N}\sum_{k=1}^{K}r_{nk}ln{\overset{ˇ}{\pi }}_{k}\right]+\left[lnC\left(\alpha_{0}\right)+\left(\alpha_{0}-1\right)\sum_{k=1}^{K}ln{\overset{ˇ}{\pi }}_{k}\right]\\ +\left[\frac{1}{2}\sum_{k=1}^{K}\left\{Dln\left(\frac{\beta_{0}}{2\pi }\right)+ln{\tilde{\Lambda }}_{k}-\frac{D\beta_{0}}{\beta_{k}}-\beta_{0}\upsilon_{k}\left({\left(m_{k}-m_{0}\right)}^{T}W_{k}\left(m_{k}-m_{0}\right)\right)\right\}+KlnB\left(W_{0},v_{0}\right)+\left(\frac{v_{0}-D-1}{2}\right)\sum_{k=1}^{K}ln{\tilde{\Lambda }}_{k}-\frac{1}{2}\sum_{k=1}^{K}v_{k}T_{r}\left(W_{0}^{-1}W_{k}\right)\right]\\ -\left[\sum_{n=1}^{N}\sum_{k=1}^{K}r_{nk}lnr_{nk}\right]-\left[\sum_{k=1}^{K}\left(\alpha_{k}-1\right)ln{\overset{ˇ}{\pi }}_{k}+lnC\left(\alpha \right)\right]\\ -\left[\sum_{k=1}^{K}\left\{\frac{1}{2}ln{\tilde{\Lambda }}_{k}+\frac{D}{2}ln\left(\frac{\beta_{k}}{2\pi }\right)-\frac{D}{2}-ℋ\left[q\left(\Lambda_{k}\right)\right]\right\}\right], \end{array}$$

where

(33) $$\begin{array}{c} \ln{\overset{ˇ}{\pi }}_{k}=E\left[\ln\pi_{k}\right]\\ B\left(W,v\right)={\left|W\right|}^{-v/2}{\left\{2^{vD/2}\pi^{D\left(D-1\right)/4}\prod_{i=1}^{D}\Gamma \left(\frac{v+1-i}{2}\right)\right\}}^{-1}\\ C\left(\alpha \right)=\frac{\Gamma \left(\hat{\alpha }\right)}{\Gamma \left(\alpha_{1}\right)\cdots \Gamma \left(\alpha_{k}\right)}\text{ and}\\ ℋ\left[\Lambda \right]=-\ln B\left(W,v\right)-\frac{\left(v-D-1\right)}{2}E\left[\ln\left|\Lambda \right|\right]+\frac{vD}{2}. \end{array}$$

In this paper, we implement the maximization of equation (32) through the iterative updates of the GMM parameters mentioned earlier.

### 3.3. Variational Mixture of Gaussians (VMGs) Routing-Based Capsule Network

Motivated by [10, 11], and [4] based on the discussions in Sections 3.1 and 3.2, we let ℒ_*n*_ and ℒ_*k*_, respectively, represent capsules at the lower and higher-level layers. Let *X*_*k|n*_ ∈ ℝ^4*x*4^ matrix represent the show of similarity between the features of a lower-level capsule *n* to a higher-level capsule *k*, with *x*_*k|n*_ ∈ ℝ^*D*^ as its vectorized version (i.e. x_*k|n*_ is a flattened vector of the matrix *X*_*k|n*_ with *D* = 16). A higher-level capsule's pose matrix *M*_*k*_ ∈ ℝ^4*x*4^ is flattened to obtain capsule *k*'*s* pose vector *μ*_*k*_ ∈ ℝ^*D*^. For ease of computations, we use the precision matrix Λ_*k*_ instead of the covariance matrix *Σ*, and use *λ*_*k*_ ∈ ℝ^*D*^ to represents the diagonal entries of Λ_*k*_. As mentioned earlier, *r*_*nk*_ represents the vector form of the routing responsibilities while *π*_*k*_ is the mixing coefficient used for a single one-hot-vector representation (1/*k*) necessary for indicating the choice of a cluster(capsule). On a larger scale, *z* is a latent variable that serves as a collection of one-hot-vectors with similar features signifying the preference of each lower-level capsule feature to a corresponding higher-level capsule Gaussian cluster of features. Finally, we compute the activation probability *a*_*n*_ to represent the likelihood that cluster *k* is activated by computing the ELBO (equation (32)) and paying a fixed cost of *β*_*a*_ as indicated in [4]. Based on the above-given discussions, we derive Algorithm 1 as the routing procedure between capsules.

### 3.4. Uncertainty Estimation

Aleatoric and epistemic uncertainties are common with neural network models. Randomness is a property that characterizes aleatoric uncertainty [21]. For this type of uncertainty, there is sufficient variability in the outcome of events as a result of a random phenomenon. Epistemic uncertainty, on the other hand, expresses the uncertainty resulting from the designer's lack of knowledge of the best design choices leading to the development of the best model. Both uncertainties together form the total uncertainty of the model. Several other methods exist for finding the total uncertainty of a model, but there is no consensus on which method is the best [25].

In this work, we experimentally determine the aleatoric and epistemic uncertainties of our model on some of the datasets. Since a deterministic model has no epistemic uncertainty [25], we determine its aleatoric uncertainty on the *in* and *out*-of-distribution data. For our Bayesian model, we determine both uncertainties.

## 4. Experiments

The experiments in this work were carried out using *PyTorch 1.7* GPU version on a 64 bit NVIDIA GeForce GTX 1060 Windows machine. Each model was trained for 100 epochs using a learning rate of 0.001, 3 routing iterations, and patience of 10,000. During training, the best model is saved to be used for inference. The code used in our implementation is a modification of the code in [11], which can be found in [26].

### 4.1. Loss Function

We adopted the spread loss in [4] as well as the negative likelihood loss as used in [11].

### 4.2. Model Architecture

Our model begins with a 2 × 2-filter convolutional layer to perform convolutions on a 32 × 32 × 1 input image with a stride of 2. This layer precedes three capsule layers and the ensuing VMG routing layers before the final class capsule layer which produces one capsule for each capsule class. Each capsule layer converts its respective filters into a 4 × 4 *p*_*i*_ capsule pose matrix and activation. The final layer broadcasts its weight matrices to produce a capsule *p*_4_ per class for each category in the dataset. Taking the filter *f* and the capsule types *p*_*i*_ produced by each capsule layer into consideration, the network for the model can be represented as [*f*, *p*_1_, *p*_2_, *p*_3_, *p*_4_]. The complete architecture is shown in Figure 1.

### 4.3. Datasets and Data Preprocessing

Three popular computer vision datasets and one health-related dataset were adopted to experimentally evaluate the methods proposed in this paper. MNIST [27] is a handwritten dataset consisting of 70,000 28 × 28 grayscale images commonly partitioned into 60,000 training and 10,000 test sets. Comparatively, this dataset is less complex but effective and very popular for testing the performance of computer vision algorithms. Fashion-MNIST [28] is another dataset obtained from 70,000 greyscale fashion products. The original partition into training and test sets is similar to MNIST. This dataset is relatively complex to MNIST. The third and most complex dataset among the three is CIFAR-10 [29]. This dataset is very challenging to most computer vision algorithms due to the presence of background as well as background objects. Each of the aforementioned datasets is made up of ten classes and was partitioned into 55000 training, 5000 validation, and 10,000 test sets.

The fourth dataset is a COVID-19 Radiography dataset [30–32] collected from four countries by a team of doctors. It consists of three classes of infected chest X-ray images and one class of healthy X-rays. This dataset is highly imbalanced and for purposes of this work, was partitioned into 16,952 training, 2,000 validation, and 4,227 test images. Even though the performance of some machine vision algorithms largely depends on extensive preprocessing to obtain high informative image data, we did not employ any of these preprocessing algorithms irrespective of the fact that digital images contain Gaussian noise introduced by the limitations of the acquisition sensor/camera during image capturing. Fortunately, there are techniques to reduce its effect [33]. However, we evaluated the model on the raw images, enabling us to understand the actual extent to which the model can recognize real-life digital images (such as the COVID-19 images) without human interference.

### 4.4. Experimental Results

The results presented in this section are from the implementation of our model (Variational Mixture of Gaussians Routing model-VMG-Routing), the baseline Multilane LBP-Gabor Capsule (ML) network [32], and the VB-Routing [11] {64, 8, 16, 16, #c} architecture; where #c is the number of output classes. However, our GPU device could not run the higher architectures of the other VB-Routing models, consequently, for those models, we reported the results from the work in [11].

#### 4.4.1. Model Learning and Convergence

The training and validation curves in Figure 2 show the proposed model's ability to learn and converge faster. For less complex images such as MNIST and Fashion-MNIST, the model converges as early as epoch 30. For relatively complex and imbalanced images such as CIFAR-10 and COVID-19 Radiography, the model attains an accuracy approximately equal to the final accuracy at epoch 90. Our VMG-Routing learns faster compared to the models in [11] which only show stability beginning from epoch 150. Fast learning and convergence are desirable attributes for image recognition systems applied in critical areas such as self-driving cars where every passing minute counts and is valuable.

Table 1 reports a comparison of the error rates of the VMG-Routing capsule and the other capsule network (CapsNet) models. Even with the moderate (shallow) size of the VMG-Routing model, it performs comparatively well with the deep and multilane models. The difference in accuracy on CIFAR-10 between the proposed VMG-Routing CapsNet and the largest model is only 1.07% with our model having an added advantage of being less computationally complex.

#### 4.4.2. Model Complexity

The VMG-Routing CapNet produced fewer parameters compared to its counterparts in the literature as can be seen in Table 2. This makes the VMG-Routing model less computationally complex and increases its potential for implementation on embedded and mobile devices that naturally have limited memory. In addition, model complexity poses a threat of overfitting [34] that ultimately leads to poor performance.

#### 4.4.3. Inference

To test the models' generalizability on unseen images, we used the trained (saved) models to perform inference, respectively, on 10,000 and 4,227 sample images from MNIST, CIFAR-10, Fashion-MNIST, and the COVID-19 Radiography datasets. A comparison of the test accuracies is reported in Table 3. The average time for each model to perform inference on the sample images is also reported in Table 3. It can be observed that the VMG-Routing model produced results that compare favorably well with the results of other state-of-the-art models.

We further performed inference on individual in-distribution images for both models to determine the level of confidence/certainty each model places on its prediction probabilities.  Figure 3 shows that the deterministic model is overconfident in its predictions (column 3) while the VMG-Routing CapsNet exercises some caution in the confidence it imposes on its predictions (column 2).

#### 4.4.4. Model Uncertainty

Daily scenarios involve decision-making influenced by the level of uncertainties/certainties prevailing at the time. Depending on the field under consideration, uncertainty estimation can be a critical part of the decision-making process. For instance, the reliability and efficacy of a deep learning model for medical applications such as Artificial Intelligence (AI) assisted surgery depends on the uncertainty with which it identifies the medical condition correctly. Bayesian methods have advantages over other neural networks as they provide the avenue to effectively model uncertainty [12]. The inability of machine learning applications to provide reliable uncertainty estimates is a potential limiting factor in their acceptability and widespread adoption for critical tasks.

To demonstrate the reliability of the uncertainty estimates of our VMG-Routing model, we present a comparison of experimental results from the prediction of both in-distribution (Figure 4) and out-of-distribution (Figure 5) images for the VMG-Routing model and the baseline deterministic ML-LBP capsule model.

We use *p*_out_ to express the aleatoric uncertainty shown by the distribution across the classes for the deterministic model. This uncertainty assumes a value of zero if a class gets a probability of one and all other classes obtain a probability of zero. Since deterministic CapsNets have fixed weights, they cannot express epistemic uncertainties [25] and will produce the same output when inference is carried on the same input image *N* times. The output of the SoftMax layer *p*_out_ (see Figure 3) sums up to one and measures the certainty (certainty = *p*_out_) of the model in its predictions. We obtain the aleatoric uncertainty of the deterministic CapsNet from the same quantity *p*_*out*_ by computing the negative log likelihood (NLL) or the entropy of the predictions.

(34) $$\begin{array}{c} \text{entropy}=-\sum_{i=0}^{\#c}p_{i}\log\left(p_{i}\right),\\ \text{aleatoric uncertainty}=NLL\\ =-\log\left(p_{\text{out}}\right), \end{array}$$

where 0 ≤ *i* < #*c* and #*c* is the number of classes in the dataset under consideration.

On the other hand, our VMG-Routing CapsNet replaces the fixed weights with Gaussian distributions giving it the ability to express both epistemic and aleatoric uncertainties in its predictions. The aleatoric uncertainty is expressed in the distributions similar to the deterministic CapsNets, except that it is based on average prediction probabilities. Meanwhile, the epistemic uncertainty is measured in the spread of the inference probabilities and is zero for a zero spread. For this scenario, *N* different multinomial conditional probability distribution $p\left(\hat{y}|x,w_{n}\right)$ conditioned on the weight distribution *w*_*n*_ are obtained out of *N* predictions on the same input image. The mean probability *p*_out_^*∗*^ is computed for each class *i* and the maximum mean conditional probability is chosen as the predicted class of the input image.

(35) $$\begin{array}{c} p_{\text{out}}^{*}=\frac{1}{N}\sum_{i=0}^{N-1}p_{{\text{out}}_{i}}, \end{array}$$

and

(36) $$\begin{array}{c} p_{\text{inf}}^{*}=\max\left(p_{\text{out}}^{*}\right). \end{array}$$

The averaging in the measure in equation (35) ensures that the epistemic uncertainty in the model is captured. Subsequently, *NLL*^*∗*^ = −log(*p*_inf_^*∗*^) is possible to compute. In addition, the uncertainty based on the entropy and total variance obtained from the averaging naturally follows from the following expressions:

(37) $$\begin{array}{c} {\text{entropy}}^{*}=-\sum_{i=0}^{\#c}p_{\text{out}}^{*}\log\left(p_{\text{out}}^{*}\right),\\ \sigma_{T}^{2}=\sum_{i=0}^{\#c}\sigma^{2}\left(p_{i}\right)=\sum_{i=0}^{\#c}\frac{1}{N}\sum_{n=0}^{N-1}{\left(p_{in}-p_{i}^{*}\right)}^{2}. \end{array}$$

Figure 5 shows the uncertainty of both models on the respective out-of-distribution images. The spread of the prediction probabilities of a given class expresses the epistemic uncertainty while the distribution across the different classes epitomizes the aleatoric uncertainty of the models [25].

Even though both models produce wrong predictions for the out-of-distribution images, the VMG-Routing CapsNet produces predictive probabilities (Figure 5, column 2) that significantly vary in the distribution and spread of the *N*=100 predictive runs. The VMG-Routing CapsNet, therefore, can express both uncertainties. On the contrary, the deterministic model cannot express epistemic uncertainty since performing *N*=100 predictive runs on the same input image produces the same probabilities (Figure 5, column 3). The ability of a model to express its uncertainty is a desirable property since it can be shown that models that produce higher uncertainties are likely to produce accurate predictions [25]. Finally, the shape of the VMG-Routing CapsNet's predictive probability distribution has some semblance to that of the Gaussian distribution which may be attributed to the model being driven by a variational mixture of Gaussians.

#### 4.4.5. Model's Ability to Extract Relevant Features

To enable us to understand and tune the VMG-Routing model for further performance improvement, we investigated the ability of the layers in the model to extract the relevant features. Through experimentation via this approach, redundant layers were eliminated, resulting in a reduction in the model size/complexity, convergence time, and excessive oscillations during training. More specifically, we visualized the output (feature maps) of the layers by feeding an input image into the trained (best saved) model. The feature maps for the various layers are shown in Figure 6. It can be observed that the layers of the model can extract the most relevant features from the input images.

#### 4.4.6. Threats to Validity

Deep Learning (DL) is capable of learning and modeling real-life scenarios when extreme care is taken, during the design and development stages, to consider all the factors that have the potential to prevent the model from achieving optimal performance. For instance, the choice of hyperparameters and their values is an important exercise that has a direct impact on the validity of the model outputs. For stochastic gradient descent (SGD)-based methods and their variants, a fraction of the dataset used for training are organized into batches whose size is relevant to the computation of the gradient. Practically, larger batch sizes reduce the quality of the model during generalization [35]. This work, therefore, sampled from 16–32 data points for the experiments as batch sizes. We also avoided the sorting of the dataset and introduced randomization of batches in a bid to prevent the possibility that a given batch will have the same labels. In addition, the learning rate controls the rate at which the model should be modified in response to the error anytime there is an update in the model weights. We chose a smaller learning rate to allow the model to learn the optimal set of weights even though this has the potential to increase training time and the risk of overfitting. Other methods for solving this include implementing a learning rate decay function which returns an updated learning rate value that drops by half every *n* number of epochs. Furthermore, nonlinear activation functions are useful for DL to effectively model real-life scenarios which are nonlinear. The choice of the appropriate activation function determines the speed of computations necessary to speed up the training process as well as the ability to reduce the likelihood of generating vanishing gradients and improve performance [36]. To introduce nonlinearity and activate the capsule, we adopted the Sigmoid activation function since it encourages unambiguous predictions with 1 or 0, plus the fact that it can return a value between 0 and 1 when used with (−*∞*, +*∞*).

Another scenario that poses a threat to the validity of the Bayesian model outputs is the covariate shift, where the distributions of training and target data are different [37]. Covariate shift may also occur due to pixelate-corrupted test data, spurious correlations, and domain shift. This problem is well pronounced with Bayesian models that make use of unconstrained Λ (covariance matrix) and is worsened when there exists linear independence in the features. In this work, we employed mean-field variational inference (MFVI) which constraints the Λ to be a diagonal matrix, limiting the effect of linear dependence in the features [38] and hence the impact of covariate shift.

## 5. Conclusion and Future Work

In this work, we proposed a capsule network based on a variational mixture of Gaussian routing to express the uncertainties associated with performing predictions on out-of-distribution data. The results show that a Bayesian capsule can be less computationally complex, converge faster, and outperform both the state-of-the-art deterministic and probabilistic models during inference. Furthermore, our work demonstrates that Bayesian capsules may have advantages over their deterministic counterparts since they have a bigger potential to exhibit transparency, credibility, reliability, and interpretability required to gain the confidence of industry players.

In the future, we intend to carry out a full investigation into Bayesian capsule interpretability in a quest to unravel the “black box” concept.

## Figures and Tables

**Figure 1:** Architecture of the proposed VMG CapsNet model.

**Figure 2:** Training/validation accuracy/loss curves for the proposed model. The model learns and converges on (b) Fashion-MNIST and (c) MNIST as early as epoch 30. Learning takes time for (a) CIFAR-10 and (d) COVID-19 Radiography images but achieves convergence at epoch 90. We notice that the model converges faster for the images that are less complex compared to CIFAR-10 and COVID-19.

**Figure 3:** Comparison of the prediction probabilities of the VMG-Routing CapsNet and the Multi-lane LBP-Gabor Capsule model on in-distribution COVID-19 and MNIST test images. These results express the certainty of each model in its prediction of the test image. Notice that the deterministic model produces higher probabilities as a way of expressing overconfidence.

**Figure 4:** Comparison of the uncertainty between the VMG-Routing and Multi-lane CapsNets on in-distribution test images. The VMG-Routing CapsNet shows uncertainty over the ML model on the MNIST dataset. On the COVID-19 dataset, the uncertainty for both models is approximately the same.

**Figure 5:** Uncertainty plots for (column 2) the VMG CapsNet on the out-of-distribution images, and (column 3) the deterministic Multilane LBP CapsNet on the same two images. The spread of the VMG CapsNet predictions demonstrates its high epistemic uncertainty on the images. On the other hand, the Multi-lane LBP CapsNet shows false confidence in its predictions as shown by the consistency with which it produces the same probabilities for the *N*  =  100 predictive runs.

**Figure 6:** Visualization of the feature maps for the layers in the VMG-Routing model. The first two rows show the MNIST input image and the outputs of each layer. The second two rows show the input from a COVID-19 Radiography image and the corresponding outputs of the filters for each layer.

**Algorithm 1:** Variational mixture of Gaussians routing.

**Table 1:** Comparison of the error rates between the VMG-Routing model and some models from the literature. (*∗*) indicates the models that our device could not implement due to memory limitations. The values reported here were thus obtained from the literature. (−) indicates unavailable values. (#c) represents the number of classes in the dataset.

Algorithm	Error rate (%)			
	CIFAR-10	Fashion-MNIST	MNIST	COVID-19 radiography
VB-routing {64, 8, 16, 16, #*c*} [11]	13.10	5.46	0.99	8.01
VB-routing*∗* {64, 16, 32, 32, #*c*} [11]	11.2 ±.09	5.61	—	—
VB-routing*∗* {64, 16, 16, 16, #*c*} [11]	12.40	5.2 ±.07	—	—
EM-routing*∗* {64, 16, 16, 16, #*c*} [4]	—	6.14	—	—
EM-routing*∗* {64, 16, 32, 32, #*c*} [4]	11.2 ±.09	—	—	—
Multi-lane LBP-gabor capsule [32]	11.43	5.17	1.00	8.04
Dynamic routing [3]	35.57	22.45	0.25	8.09
VMG-routing {32, 4, 8, 8, #*c*} (**ours**)	12.19	5.38	1.00	7.01

**Table 2:** Comparison of the number of parameters generated by each model. The VMG-Routing model produced the least number of parameters with the ML producing the largest number of parameters. (*∗*) indicates the models that our device could not implement due to memory limitations. The values reported here were thus obtained from the literature. (−) indicates unavailable values. (#c) represents the number of classes in the dataset.

Algorithm	Number of parameters			
	CIFAR-10	Fashion-MNIST	MNIST	COVID-19 radiography
VB-routing {64, 8, 16, 16, #*c*}	145 K	145 K	145 K	120 K
VB-routing*∗* {64, 16, 32, 32, #*c*}	323 K	323 K	—	—
VB-routing*∗* {64, 16, 16, 16, #*c*}	172 K	172 K	—	—
EM-routing*∗* {64, 16, 16, 16, #*c*}	—	323 K	—	—
EM-routing*∗* {64, 16, 32, 32, #*c*}	323 K	—	—	—
Multi-lane LBP-gabor capsule	4.10 M	4.10 M	4.10 M	3.70 M
Dynamic routing	9.3 M	8.2 M	8.2 M	9.8 M
VMG-routing {32, 4, 8, 8, #*c*} (**ours**)	14 K	15.5 K	14 K	10.2 K

**Table 3:** Results of testing on 10,000 sample images of MNIST, CIFAR-10, and Fashion-MNIST dataset. 4,227 samples were used for testing the models on the COVID-19 Radiography dataset.

Algorithm	MNIST (%)	CIFAR-10 (%)	Fashion-MNIST (%)	COVID-19 Radiography	Average time
VB-routing {64, 8, 16, 16, #*c*}	98.53	85.06	92.97	90.92%	30 s, 14 ms
Multi-lane LBP-gabor capsule	98.89	86.97	94.00	91.09%	18 s, 25 ms
Dynamic routing	99.21	65.11	76.32	90.02%	20 s, 11 ms
VMG-routing {32, 4, 8, 8, #*c*} (**ours**)	98.96	86.82	93.71	92.15%	15 s, 23 ms

## Data Availability

The data used to support the findings of this study can be accessed in the following repositories: 1. http://yann.lecun.com/exdb/mnist/ 2. https://www.cs.toronto.edu/∼kriz/cifar.html 3. https://www.kaggle.com/datasets/zalando-research/fashionmnist 4. https://www.kaggle.com/datasets/preetviradiya/covid19-radiography-dataset.
